This article has been retracted.

# Clinical Value of Cytokine Assay in Diagnosis and Severity Assessment of Lung Cancer

**DOI:** 10.1155/2022/4641600

**Published:** 2022-08-09

**Authors:** Jin Ma, Shumin Zhu, Zining Liu, Yafei Mao, Xinyuan Li, Lili Dai, Xiaojie Zhao, Congzhen Wei, Jinfeng Liu, Yulan Geng

**Affiliations:** ^1^Laboratory, The Third Hospital of Hebei Medical University, Shijiazhuang 050051, Hebei Province, China; ^2^Laboratory, The First Hospital of Hebei Medical University, Shijiazhuang 050030, Hebei Province, China

## Abstract

**Purpose:**

To investigate the clinical value of interleukin 2 (IL-2), interleukin 4 (IL-4), interleukin 6 (IL-6), interleukin 10 (IL-10), tumor necrosis factor *α* (TNF-*α*), and interferon-*γ* (IFN-*γ*) in diagnosis and severity assessment of lung cancer.

**Methods:**

In this observational study, 50 physical examination healthy subjects were included in the control group and 100 lung cancer patients were included in the study group. In the study group, 53 cases with pleural effusion were subgrouped to the pleural effusion group (*n* = 53), while 47 patients were assigned to the nonpleural effusion group (*n* = 47). Plasma cytokines IL-2, IL-4, IL-6, IL-10, TNF-*α*, IFN-*γ*, and Acute Physiology and Chronic Health Evaluation II (APACHE II) scores of all eligible subjects were collected and compared.

**Results:**

The study group showed significantly higher levels of plasma cytokines IL-2, IL-4, IL-6, IL-10, TNF-*α*, and IFN-*γ* versus healthy subjects (*P* < 0.05). Deterioration of lung cancer was associated with increased plasma cytokine levels and APACHE II scores. The combination assay of the above plasma cytokines showed significantly better diagnostic efficacy for lung cancer versus the single assay of the cytokines. Dead patients had higher plasma cytokine levels versus survived patients. The accuracy of plasma IL-2, IL-4, IL-6, IL-10, TNF-*α*, and IFN-*γ* levels in the severity assessment of lung cancer was comparable with that of the APACHE II scale.

**Conclusion:**

The plasma cytokines IL-2, IL-4, IL-6, IL-10, TNF-*α*, and IFN-*γ* are effective markers for the diagnosis of lung cancer. The combined assay contributes to the early diagnosis of lung cancer patients, and the persistent elevation of cytokines suggests an increased risk of death in lung cancer patients, so the detection of cytokine levels facilitates the severity assessment of lung cancer.

## 1. Introduction

Due to the impact of the poor living environment such as urban industrialized pollution, the prevalence and mortality rate of lung cancer in China show a rising trend year-by-year [1, 2]. Lung cancer includes small cell lung cancer (SCLC) and nonsmall cell lung cancer (NSCLC), and the 5-year overall survival for patients with NSCLC and SCLC remains at a low level due to the absence of effective early diagnostic methods and tumor recurrence [3, 4]. Therefore, early diagnosis is of great significance to enhance the prognosis of patients. Serum tumor markers provide referential evidence for tumor diagnosis, treatment efficacy, and prognosis, but their sensitivity is considered unsatisfactory for early stage lung cancer. Previous research has reported the role of immunomodulatory cytokines in tumor growth and metastasis [5]. Cytokines are involved in the normal immune homeostasis of the body and play a vital role in regulating tumorigenesis and progression, treatment prognosis, and antitumor immune regulation. Important cytokines in the human body include interleukin-1*β* (IL-1*β*), IL-2, IL-4, IL-6, IL-10, TNF-*α*, and IFN-*γ* and transforming growth factor (TGF)-*β*1 [6, 7]. Some of these cytokines may be effective in killing tumor cells, regulating immune response, promoting cell proliferation, stimulating hematopoietic tissue, counteracting the side effects of chemotherapy and radiotherapy, improving prognosis, and prolonging patient survival [8]. The role of cytokines in tumor growth and metastasis has been widely recognized, but with few studies in diagnosis [9]. In the present study, 100 patients with lung cancer and 50 healthy individuals were identified as research subjects to investigate the value of cytokine assay in diagnosis and severity assessment of lung cancer for prognosis judgment and stratified management of patients.

## 2. Materials and Methods

### 2.1. Research Subjects

Between January 2018 and December 2020, 100 patients with a first clinical diagnosis of lung cancer were recruited as the study group. They were assigned to a pleural effusion group or a nonpleural effusion group according to the presence of pleural effusion. 50 healthy individuals were included in the control group. Ethical approval for this study was obtained from Ethics Committee of the First Hospital of Hebei Medical University, No. 10797/1.

### 2.2. Inclusion and Exclusion Criteria

Patients who were diagnosed with nonsmall cell lung cancer by histopathology or cytology; with pleural effusion confirmed by cytological examination in the pleural effusion group; with cancer in stage IIIB or IV; with Eastern Cooperative Oncology Group (ECOG) performance status of 0, 1, or 2; and aged 18–80 years were included.

Patients with an ECOG performance status of 3 or worse; with a history of congestive heart failure, myocardial infarction, or life-threatening arrhythmia; and with other tumor types or other subtypes of lung cancer were excluded.

### 2.3. Methods

2 ml of venous blood was collected from all eligible subjects, and 2 ml of pleural effusion was collected from the patients of the effusion group, and the levels of plasma cytokines IL-2, L-4, IL-6, IL-10, TNF-*α*, and IFN-***γ*** were determined with a flow cytometer. The flow cytometer NAVIOS was supplied by Beckman, USA, and the cytokine detection reagents, calibrators, and quality control products were provided by Jiangxi Saiki Biotechnology Co.

### 2.4. APACHE II Score

All lung cancer patients were scored on admission by the APACHE II scale to assess the severity of the disease.

### 2.5. Statistical Analysis

SPSS 25.0 statistical software was used for data analyses. The measurement data are expressed as (mean ± SD) and analyzed using the *t*-test for intergroup comparison. The count data are expressed as rates (%) and analyzed using the chi-square test for intergroup comparison. Differences were considered statistically significant at *P* < 0.05. Logistic regression models were developed from the combined diagnostic data, and receiver operating characteristic curves (ROC) were applied to assess diagnostic efficacy and were represented using the area under the curve.

## 3. Results

### 3.1. Baseline Data

There were 53 cases in the effusion group including 27 males and 26 females with a mean age of 65 ± 11.75 years, and 47 cases in the no effusion group including 23 males and 24 females with a mean age of 62 ± 13.38 years. All eligible subjects in the three groups showed similar baseline characteristics (*P* > 0.05). The patients in the pleural effusion group showed higher APACHE II scores than those in the nonpleural effusion group, indicating more severe conditions of lung cancer in patients with pleural effusion versus those without pleural effusion (*P* < 0.05) (Table 1).

### 3.2. Plasma Cytokine Levels and APACHE II Score

The eligible patients showed significantly higher levels of plasma cytokines IL-2, IL-4, IL-6, IL-10, TNF-*α*, and IFN-*γ* versus healthy subjects (*P* < 0.05). Deterioration of lung cancer was associated with increased plasma cytokines and elevated APACHE II scores (Table 2).

### 3.3. Efficacy of Plasma Cytokines in the Diagnosis of Lung Cancer

The combination diagnostic model equation of cytokines was Logit (*p*) = 0.021IL-2 + 0.358IL-4 + 0.698IL-6 + 1.132IL-10 + 1.0151.145TNF-*α* + 0.894FN-*γ*—2.26. The combination assay of the above plasma cytokines had significantly better diagnostic efficacy for lung cancer versus the single assay of the cytokines, with the area under the ROC curve being 0.977, 0.891, 0.887, 0.885, 0.897, 0.903, and 0.867 (Table 3).

### 3.4. Plasma Cytokine Levels of Dead or Survived Patients

There were 17 cases of death among all 100 eligible lung cancer patients. Dead patients showed higher plasma cytokine levels versus survived patients (Table 4).

### 3.5. Accuracy of Plasma Cytokines and APACHE II Scores in Predicting the Risk of Death in Lung Cancer Patients

The predictive values of plasma cytokines IL-2, IL-4, IL-6, IL-10, TNF-*α*, and IFN-*γ* alone for the mortality of lung cancer were 17.65%, 17.65%, 23.53%, 17.65%, 23.53%, and 17.65%, respectively, and the predictive value of the combination of the six cytokines for the mortality of lung cancer reached 47.06% (*P* < 0.05). The predictive value of the combined assay of the six cytokines for lung cancer death was comparable to that of the APACHE II score (*P* > 0.05). The accuracy of IL-2, IL-4, IL-6, IL-10, TNF-*α*, and IFN-*γ* in predicting the risk of death from lung cancer was 62.44%, 65.65%, 68.15%, 66.28%, 67.98%, and 66.65%, respectively. The accuracy of the combined application of the six in the prediction of the risk of death from lung cancer reached 84.37% (*P* < 0.05) and was similar to that of APACHE II scores (*P* > 0.05) (Table 5).

## 4. Discussion

With the exacerbation of environmental problems, the incidence of lung cancer in China has shown a trend of increase. Despite the continuous medical advances such as targeted drug therapy and monoclonal immunotherapy in the treatment of lung cancer, lung cancer patients still suffer a poor prognosis and survival quality [10], which necessitates effective early diagnosis and treatment methods for the disease. Data published by the World Health Organization showed the incidence rate and the mortality rate of lung cancer in China in 2020 were 17.9% and 23.8%, ranking first among all malignant tumors [11]. Carcinoembryonic antigen (CEA), squamous cell carcinoma antigen (SCC), neuron-specific enolase (NSE), glycoantigen 125 (CA125), cytokeratin-19 fragment (CYFRA21-1), and progranulin-releasing peptide precursor (proGRP) are widely used tumor markers for the screening or diagnosis of lung squamous, adenocarcinoma, and small cell carcinoma in clinical practice [12]. Nonetheless, the assay of these indices in lung cancer diagnosis is associated with good specificity but low sensitivity, which may lead to false positives [13].

The cytokines IL-6, IL-10, TNF-*α*, and IFN-*γ* have been reported to show good potential in the diagnosis and prognosis of tumors [14]. IL-2 is an interleukin that is involved in immune memory and autoimmune diseases, but its use in immunotherapy remains contentious. The results in the present study showed significantly higher IL-2 levels in lung cancer patients than those of the healthy subjects. The polymorphism of IL-4 VNTR may contribute to the development of lung cancer. IL-6 is associated with the production of lung cancer cells, postoperative recovery, quality of survival, and disease malignancy, and it inhibits the antitumor immune response ability of normal human cells, contributing to further development of lung cancer. IL-10 promotes the phagocytosis of mononuclear macrophages, the expression of various receptors [15], and the activation and proliferation of CD8+ T cells, thereby enhancing the body's antitumor capacity and inhibiting the secretion of proinflammatory cytokines. TNF-*α* mediates the body's autoimmune response, but its persistent release may aggravate the body's pathological damage and promote tumor proliferation. High levels of TNF-*α* in tumor patients are associated with a higher risk of metastasis and postoperative recurrence. IFN-*γ* promotes MHC molecule expression and antigen presentation, facilitates Th1 cell differentiation, and inhibits Th2 cell differentiation [16], providing antitumor, antigen presentation, and immunomodulatory effects in the organism. The coactivity of TNF-*α* and IFN-*γ* enhances the expression of immunomodulatory proteins, but the relationship between these cytokines and tumor progression is poorly understood, and research on the relationship between interleukins and disease severity and their role in the pathogenesis of lung cancer is marginally explored.

The results of the present study showed that all eligible patients showed significantly higher levels of plasma cytokines IL-2, IL-4, IL-6, IL-10, TNF-*α*, and IFN-*γ* versus healthy subjects (*P* < 0.05). Deterioration of lung cancer was associated with increased plasma cytokines and APACHE II scores. The combination assay of the above plasma cytokines had significantly better diagnostic efficacy for lung cancer versus the single assay of the cytokines [17], with the area under the ROC curve being 0.977, 0.891, 0.887, 0.885, 0.897, 0.903, and 0.867, indicating the combined cytokines assay could be effective in the early diagnosis of lung cancer. In addition, the results of this study showed that dead patients were associated with higher plasma cytokine levels versus survived patients [16] and that the predictive value of the combined judgment of the six cytokines for lung cancer death was comparable to that of the APACHE II score. The APACHE II score is clinically used to classify the condition of critically ill patients and to assess their prognosis, and it consists of categories A (acute physiology score (APS)), B (age score), and C (chronic health status score), which can be used quantitatively and dynamically for severity assessment of the patient's condition, and the score is inversely proportional to the prognosis [18]. The similar predictive value between the APACHE II score and the joint assay of the cytokines suggests the feasibility of the mortality assessment using the levels of plasma cytokines IL-2, IL-4, IL-6, IL-10, TNF-*α*, and IFN-*γ* measurements [19].

## 5. Conclusion

The plasma cytokines IL-2, IL-4, IL-6, IL-10, TNF-*α*, and IFN-*γ* are effective markers for the diagnosis of lung cancer. The combined assay contributes to the early diagnosis of lung cancer patients, and the persistent elevation of cytokines suggests an increased risk of death in lung cancer patients, so the detection of cytokine levels facilitates the severity assessment of lung cancer [20] and the reduction of mortality rates of lung cancer. In-depth studies of the mechanism and regulation of plasma cytokines in the pathological changes in lung cancer will be conducted in the future to provide new ideas for the clinical diagnosis and treatment of lung cancer.

## Figures and Tables

**Table 1:** Comparison of baseline data.

Groups	*n*	Gender		Age (year)	APACHE II scores (points, $\bar{x}$ ± *s*)
		Male	Female		
Control group	50	26	24	60.43 ± 10.33	—
Nonpleural effusion group	47	23	24	62.15 ± 13.38	12.4 ± 3.9
Pleural effusion group	53	27	26	65.56 ± 11.75	19.97 ± 3.82

**Table 2:** Plasma cytokine levels and APACHE II score.

Groups	*n*	IL-2 (pg/ml)	IL-4 (pg/ml)	IL-6 (pg/ml)	IL-10 (pg/ml)	TNF-*α* (pg/ml)	IFN-*γ* (pg/ml)	APACHE II scores (points, $\bar{x}$ ± *s*)
Control group	50	2.05 ± 1.24	1.14 ± 0.98	1.04 ± 0.86	1.33 ± 1.11	0.96 ± 0.65	1.58 ± 1.12	—
Nonpleural effusion group	47	15.22 ± 3.14^a^	19.85 ± 2.06^a^	18.98 ± 2.45^a^	16.98 ± 3.87^a^	23.47 ± 2.25^a^	11.64 ± 2.09^a^	12.4 ± 3.9
Pleural effusion group	53	39.59 ± 6.43^ab^	65.63 ± 15.36^ab^	106.28 ± 20.92^ab^	78.48 ± 12.15^ab^	95.71 ± 18.33^ab^	68.91 ± 11.37^ab^	19.97 ± 3.82

^a^ *P* < 0.05, comparison between the pleural effusion group and the healthy controls; ^b^*P* < 0.05, comparison between the pleural effusion group and the nonpleural effusion group; — indicates no available data for this item.

**Table 3:** Confidence interval of the area under the ROC curve for IL-2, IL-4, IL-6, IL-10, TNF-*α*, and IFN-*γ* and combined regression for the diagnosis of lung cancer.

Variables	Area under the curve	Standard errors	Progressive sig	95% confidence interval
IL-2	0.891	0.023	0.000	0.839–0.942
IL-4	0.887	0.033	0.000	0.778–0.891
IL-6	0.885	0.028	0.000	0.835–0.939
IL-10	0.897	0.038	0.000	0.842–0.945
TNF-i	0.903	0.029	0.000	0.836–0.979
IFN-*γ*	0.867	0.026	0.000	0.825–0.928
Logit (IL-2+IL-4+IL-6+IL-10+TNF-*α*+IFN-*γ*)	0.977	0.031	0.000	0.912–0.998

**Table 4:** Plasma cytokine levels of dead or survived patients ($\bar{x}$ ± *s*).

Groups	n	IL-2 (pg/ml)	IL-4 (pg/ml)	IL-6 (pg/ml)	IL-10 (pg/ml)	TNF-*α* (pg/ml)	IFN-*γ* (pg/ml)
Survived patients	83	22.33 ± 4.75	32.14 ± 9.98	49.38 ± 12.15	30.22 ± 9.25	58.26 ± 11.76	32.82 ± 10.21
Dead patients	17	53.22 ± 2.01	81.62 ± 20.58	162.85 ± 36.19	92.43 ± 23.52	123.45 ± 35.69	88.85 ± 26.12
*P* value		<0.01	<0.01	<0.01	<0.01	<0.01	<0.01

**Table 5:** Accuracy of plasma cytokines and APACHE II scores in predicting the risk of death in lung cancer patients.

Items	IL-2	IL-4	IL-6	IL-10	TNF-*α*	IFN-*γ*	Combined detection	APACHE II
Mortality rate (%)	17.65 (3/17)	17.65 (3/17)	23.53 (4/17)	17.65 (3/17)	23.53 (4/17)	17.65 (3/17)	47.06 (8/17)	52.94 (9/17)
Accuracy (%)	62.44	65.65	68.15	66.28	67.98	66.65	84.37	85.77

## Data Availability

The data used to support this study are available from the corresponding author upon request.
